This article has been retracted.

# Association of cord blood asprosin concentration with atherogenic lipid profile and anthropometric indices

**DOI:** 10.1186/s13098-022-00844-7

**Published:** 2022-05-18

**Authors:** Hanan Khudhair Hussein, Malik Aubead, Hamzah H. Kzar, Yasir Salam Karim, Ali H. Amin, Moaed E. Al-Gazally, Tousief Irshad Ahmed, Mohammed Abed Jawad, Ali Thaeer Hammid, Abduladheem Turki Jalil, Yasser Fakri Mustafa, Marwan Mahmood Saleh, Hafez Heydari

**Affiliations:** 1 College of Medicine, University of Babylon, Babil, Iraq; 2 Department of Obstetrics and Gynecology, Hammurabi College of Medicine, University of Babylon, Babil, Iraq; 3 Veterinary Medicine College, Al-Qasim Green University, Al-Qasim, Iraq; 4 Al-Manara College For Medical Sciences, Maysan, Iraq; 5 Deanship of Scientific Research, Umm Al-Qura University, Makkah, Saudi Arabia; 6 Zoology Department, Faculty of Science, Mansoura University, Mansoura, Egypt; 7 College of Medicine, University of Al-Ameed, Karbala, Iraq; 8 Department of Biochemistry, SKIMS, Srinagar, J&K India; 9 Al-Nisour University College, Baghdad, Iraq; 10 Computer Engineering Techniques, Faculty of Information Technology, Imam Ja’afar Al-Sadiq University, Baghdad, Iraq; 11 Faculty of Biology and Ecology, Yanka Kupala State University of Grodno, 230023 Grodno, Belarus; 12 College of Technical Engineering, The Islamic University, Najaf, Iraq; 13 Department of Pharmaceutical Chemistry, College of Pharmacy, University of Mosul, Mosul, 41001 Iraq; 14 Department of Biophysics, College of Applied Sciences, University Of Anbar, Ramadi, Iraq; 15 Non-Communicable Diseases Research Center, Sabzevar University of Medical Sciences, Sabzevar, Iran

**Keywords:** Asprosin, Lipid profile, Umbilical cord blood, Triglyceride, Cholesterol

## Abstract

**Background:**

Elevated lipids in umbilical cord blood affect fetal programming, leading to a higher risk of developing cardiovascular disease in later life. However, the causes of changes in the lipid profile of umbilical cord blood are not clear yet. This study aimed for the first time to determine the association of asprosin concentration with TAG, TC, HDL-C, LDL-C concentrations and TAG/HDL-C, TC/HDL-C, LDL-C/HDL-C and non-HDL-C/HDL-C ratio in umbilical cord blood as well as newborn anthropometric indices. This cross-sectional study was based on 450 mother- newborn pairs of a birth cohort study in Sabzevar, Iran. Multiple linear regression was used to estimate the association of lipid concentration and lipid ratios as well as birth weight (BW), birth length (BL), head circumference (HC) and chest circumference (CC) with asprosin in cord blood samples controlled for the relevant covariates.

**Result:**

In fully adjusted models, each 1 ng/mL increase in asprosin was associated with 0.19 (95% CI 0.06, 0.31, P < 0.01), 0.19 (95% CI 0.10, 0.29, P < 0.01), 0.17 (95% CI 0.09, 0.25, P < 0.01), 0.17 (95% CI 0.09, 0.25, P < 0.01), 0.01 (95% CI 0.00, 0.013, P < 0.01), 0.01 (95% CI 0.01, 0.01, P < 0.01), 0.01 (95% CI 0.01, 0.01, P < 0.01) and 0.01 (95% CI 0.01, 0.01, P < 0.01) increase in TAG, TC, LDL-C, TAG/HDL-C, TC/HDL-C, LDL-C/HDL-C and non-HDL-C/HDL-C ratio respectively. Moreover, higher asprosin levels was positively associated with newborn BW, BL, HC and CC; however, these associations were not statistically significant.

**Conclusion:**

Overall, our findings support the positive association between cord asprosin concentration and the development of atherogenic lipid profile in newborns. Further studies are needed to confirm the findings of this study in other populations.

## Introduction

Coronary vascular disease (CVDs) is the leading cause of mortality in the world, accounting by 31.5% of all global death [1]. Atherosclerosis is the most common cause of CVDs, including ischemic heart disease, heart failure, and peripheral arterial disease [2, 3]. The atherogenic processes involved in CVDs pathogenesis begin in the intrauterine environment during fetal development and then gradually progress in subsequent years [4]. By detecting CVDs lipid risk factors including Apo A1, Apo B and atherogenic index in the umbilical cord blood of the term newborns, it is possible to recognize newborns at a higher risk for CVDs in the future [5].

The causes of changes in lipid metabolism of umbilical cord blood are not completely known. Still, there is some evidence that maternal adiposity status and adipokines (including resistin and leptin) may play an active role in regulating fetal lipid profile [6–13]. Asprosin, a novel adipokine identified by Omre et al*.*, is secreted in response to starvation from adipocytes and promotes rapid releases of glucose from the liver cells [14]. The association between circulating asprosin and lipids metabolism has been identified [15, 16]. Asprosin was positively correlated with LDL-c, APOB, APOE and TAG concentrations and negatively correlated with HDL-C concentration [15–18]. Therefore, it can be speculated that asprosin may be involved in a process that develops an atherogenic lipid profile in umbilical cord blood. To the best of our knowledge, there is no study on the association of asprosin and umbilical cord blood lipid profile. Therefore, this study aimed to investigate the relationship between umbilical cord blood asprosin with lipid profile and newborn anthropometric indices. Besides, the relationship between umbilical asprosin with different lipid ratios as predictors of CVDs has been studied.

## Material and methods

### Study population

This study was conducted from June 2018 to August 2018 at the Mobini Hospital in Sabzevar (a town in the Khorasan-Razavi province), Iran. We enrolled 450 healthy pregnant women recruited to the hospital for their delivery based on our inclusion/exclusion criteria. The inclusion criteria were mothers with a normal term of pregnancy (37–42 weeks of gestation), normal singleton pregnancies, normal vaginal delivery, normal lipid profile, self-report of no hypertension, preeclampsia, diabetes, and gestational diabetes. The exclusion criteria included intrauterine fetal growth restriction, fetal structural abnormalities, and drug intake that affects metabolism. It should be noted that the inclusion/exclusion criteria were detected through self-reports and medical records of participants. The project was approved by the Clinical Research Ethical Committee (IR.MEDSAB.REC.1397.012) of Sabzevar University of Medical Sciences and all participants signed the informed consent form before to enrollment.

### Cord blood collection and biochemical assessments

Cord blood samples were collected from the umbilical cord vein in serum separator tubes with a clot activator at delivery time. Sera were separated, aliquoted and stored at -80 until subsequent analysis. TAG, HDL-C, and TC were measured using an automated analyzer (Biotecnica, BT 1500, Rome, Italy) and commercial kits (P.L:38,231,049, Pars Azmoon, Tehran, Iran) by enzymatic colorimetric methods. LDL-C concentration was calculated using the Friedewald equation. Asprosin concentration was quantified by enzyme-linked immunosorbent assay (ELISA) using a commercially available kit according to manufacture instructions (Cat.No: CK-E91570, EASTBIOPHARM, China). Asprosin concentration was reported in ng/mL. The limit of detection (LOD) was 0.34 ng/mL. The intra-assay and interassay coefficients of variation were < 10% and < 12%, respectively.

### Statistical analyses

#### Main analysis

All statistical analyses were performed using Stata version 15 software (Stata Corp LP, College Station, Texas). The Shapiro–Wilk test and P-P plot tested the distribution of data. Data normally distributed were shown as mean ± SD and data with skewed distribution were shown as median (interquartile range (IQR)).

Multiple regression models were used to investigate the association of umbilical asprosin concentration and lipid profile and anthropometric indices. Models were further adjusted for a *priori* of the selected variables: maternal age and pre-pregnancy BMI, parity, gestational age at delivery, environmental tobacco exposure at home during pregnancy (Yes/No) and two household socioeconomic status (SES) indicators as well as two neighborhood SES indicators. Maternal education (no education, primary school, secondary school or university) and income (15 million, 15–30 million and more than 30 million riyals) were used as household SES indicators, and illiterate adults and unemployment percentages per census tract based on the last census of Iran (2016) were used as neighborhood SES indicators. Regression coefficients were reported for each 1 ng/ml increase in asprosin concentration. A significant level of 0.05 was used for all statistical analyses.

#### Sensitivity analysis

Asprosin is introduced as a fasting-induced hormone and the level of asprosin in cord blood may be significantly determined by the glucose concentration [19]. Therefore we further adjusted our models for umbilical blood glucose. Moreover, we further adjusted our models with the mother's lipid profile during pregnancy.

## Results

### Descriptive statistics

The descriptive statistics of the participants are presented in Table 1. The mean (standard deviation (SD)) age of mothers was 27.65 (5.36) years. Of the 450 newborns included in our study, 225 (50%) were male. The median (IQR) of umbilical TAG, TC, LDL-C, HDL-C, were 29.9 (26.9), 60.4 [27], 23.28 (21.48), 28.2 (12.5) mg/dL, respectively. Moreover, the median (IQR) for TAG/ HDL-C, TC /HDL-C, and Non-HDL-C/HDL-C were 1.15 (1.18), 2.01 (0.766) and 1.01 (0.76), respectively. The median (IQR) of umbilical asprosin was 30.44 (19.08) ng/mL. No significant differences were observed in asprosin concentration as well as lipid profile between male and female newborns (P-value > 0.05). The median (IQR) for birth weight (BW), birth length (BL), head circumference (HC) and chest circumference (CC) were 3250 (550) gr, 51 (3) cm, 35 (2) cm and 33 (3) cm, respectively.

**Table 1:** Descriptive statistics of participants and lipid profile

Parameter	Discription
Maternal characteristics	
Age (year); mean (SD)	27.7 (5.4)
Pre-pregnancy BMI (kg/m^2^); Median (IQR)	24.6 (5.69)
Parity; Median (IQR)	2 (1)
Gestational age (day); Median (IQR)	278 (12)
Birth weight (gr); Median (IQR)	3250 (550)
Birth length (cm); Median (IQR)	51 (3)
Head circumference (cm); Median (IQR)	35 (2)
Chest circumference (cm); Median (IQR)	33 (3)
Education	
No education/ primary school; N (%)	169 (37.6)
Secondary school education; N (%)	212 (47.1)
University degree or higher; N (%)	69 (15.3)
Self-reported tobacco exposure at home	
Yes; N (%)	81 (18.0)
No; N (%)	369 (82.0)
Income	
≥ 15 million Rials; N (%)	221 (49.1)
15 to 30 million Rials; N (%)	100 (22.2)
30 ≤ million Rials; N (%)	79 (17.5)
Illiterate percent per census tract (%); Median (IQR)	25.38 (17.5)
Unemployed percent per census tract (%); Median (IQR)	6.91 (5.1)
TAG (mg/dl); Median (IQR)	29.9 (26.9)
TC (mg/dl); Median (IQR)	60.4 (28)
HDL-C (mg/dl); Median (IQR)	28.2 (12.5)
LDL-C (mg/dl); Median (IQR)	23.28 (21.48)
Non-HDL-C (mg/dl); Median (IQR)	30.8 (21)
TC/HDL-C; Median (IQR)	2.01 (0.76)
TAG/HDL-C; Median (IQR)	1.15 (1.18)
LDL-C/HDL-C; Median (IQR)	0.78 (0.67)
Non-HDL-C/HDL-C; Median (IQR)	1.01 (0.76)
Asprosin (ng/mL); Median (IQR)	30.44 (19.08)

### Association with anthropometric indices

The results of the relationship between umbilical cord blood concentration of asprosin and BW, BL, HC and CC are presented in Table 2. In crude and adjusted models, higher levels of cord blood asprosin were positively associated with BW, BL, HC and CC as well as gestational age at delivery; however, these associations were not statistically significant.

**Table 2:** Association of cord blood asprosin concentration and anthropometric indices

Anthropometric indices	Model	β-coefficient (95% CI)	P value
Birth weight	Crude	0.64 (−1.21, 2.50)	0.49
	Adjusted	0.39 (−1.55, 2.32)	0.69
Birth length	Crude	0.01 (−0.01, 0.02)	0.42
	Adjusted	0.00 (−0.01, 0.02)	0.59
Head circumference	Crude	0.00 (−0.01, 0.01)	0.74
	Adjusted	0.00 (−0.01, 0.01)	0.52
Chest circumference	Crude	0.02 (−0.03, 0.07)	0.39
	Adjusted	0.01 (−0.06, 0.07)	0.29
Gestational age at delivery*	Crude	0.03 (−0.01, 0.06)	0.13
	Adjusted	0.02 (−0.02, 0.06)	0.24

Adjusted for Age of mother, BMI of mother before pregnancy, Number of pregnancies, Gestational age, Percent of illiterate per census tract, Percent of unemployment per census tract, Paternal education, Maternal education, Income and Tobacco exposure at home. The regression coefficient was reported based on 1 ng/mL increase in asprosin concentration

*CI* confidence interval

^*^Adjusted for above covariates except for Gestational age

### Association with lipid biomarkers

The association of asprosin concentration and lipid profile are presented in Table 3. In fully adjusted models increase in umbilical asprosin concentration was associated with increase in umbilical TAG, TC, LDL-C levels as well as TAG/HDL-C, TC/HDL-C, LDL-C/HDL-C and non-HDL-C/HDL-C ratio. Each 1 ng/ml increase in asprosin was associated with 0.19 mg/dL (95% CI 0.06, 0.31, P < 0.01), 0.19 mg/dL (95% CI 0.10, 0.29, P < 0.01), 0.17 mg/dL (95% CI 0.09, 0.25, P < 0.01), 0.17 (95% CI 0.09, 0.25, P < 0.01), 0.01 (95% CI 0.00, 0.01, P < 0.01), 0.01 (95% CI 0.01, 0.01, P < 0.01), 0.008 (95% CI 0.01, 0.01, P < 0.01) and 0.01 (95% CI 0.01, 0.01, P < 0.01) increase in TAG, TC, LDL-C, TAG/HDL-C, TC/HDL-C, LDL-C/HDL-C and non-HDL-C/HDL-C ratio respectively. The association of asprosin concentration and HDL-C concentration was not statistically significant (P-value = 0.43).

**Table 3:** Linear regression for cord asprosin concentration and change in lipid profile in newborns

		β-coefficient (95% CI)	P_value
Lipid profile			
TAG	Crude	0.19 (0.08, 0.3)	< 0.01
	Adjusted	0.19 (0.07, 0.32)	< 0.01
TC	Crude	0.19 (0.11, 0.28)	< 0.01
	Adjusted	0.20 (0.10, 0.29)	< 0.01
LDL-C	Crude	0.17 (0.10, 0.24)	< 0.01
	Adjusted	0.18 (0.10, 0.26)	< 0.01
HDL-C	Crude	−0.02 (−0.06, 0.02)	0.36
	Adjusted	−0.02 (−0.06, 0.03)	0.43
Lipid ratio			
TAG/HDL-C	Crude	0.01 (0.00, 0.01)	< 0.01
	Adjusted	0.01 (0.00, 0.01)	< 0.01
TC/HDL-C	Crude	0.01 (0.01, 0.01)	< 0.01
	Adjusted	0.01 (0.01, 0.01)	< 0.01
LDL-C/HDL-C	Crude	0.01 (0.01, 0.01)	< 0.01
	Adjusted	0.01 (0.01, 0.01)	< 0.01
Non-HDL-C/HDL-C	Crude	0.01 (0.01, 0.01)	< 0.01
	Adjusted	0.01 (0.01, 0.01)	< 0.01

Adjusted for Age of mother, BMI of mother before pregnancy, Number of pregnancies, Gestational age, Percent of illiterate per census tract, Percent of unemployment per census tract, Paternal education, Maternal education, Income and Tobacco exposure at home. The regression coefficient was reported based on 1 ng/mL increase in asprosin concentration

*CI* confidence interval

### Sensitivity analysis

The results of adjusted our models for umbilical blood glucose and mother's lipid profile on the association of asprosin concentration with anthropometric indices and umbilical lipid profile showed no notable differences in the main results in terms of significance and direction (data not shown).

## Discussion

To the best of our knowledge, this is the first study on the relationship between asprosin concentration with some anthropometric indices (e.g., HC and CC) and lipid profile in cord blood samples. We observed that serum asprosin concentration was positively associated with TAG, TC, LDL-C concentrations and TAG/HDL-C, TC/HDL-C, LDL-C/HDL-C and non-HDL-C/HDL-C ratio in umbilical cord blood. However, we did not find any significant association with HDL-C concentrations in umbilical cord blood. Moreover, there was a positive but not statistically significant association between asprosin levels and anthropometric indices.

### Interpret the results

We did not find a study on the association of asprosin concentration and lipid profile in cord blood; therefore, it is impossible to compare our results with other studies. However, several studies have examined the association of serum asprosin concentrations and lipid profile in adults. Wang et al. 2018 showed that serum concentrations of asprosin were positively correlated with TAG concentrations. They also reported that asprosin concentrations were negatively correlated with HDL-C concentrations [20]. Moreover, the association of serum concentration of asprosin and HDL-C has been reported in a study by Long et al. [16]. The studies by Whang et al. 2018 and Zhang et al*.* 2019 reported there was no statistically significant association between serum concentrations of asprosin and LDL-C [15, 20]. However, Li et al*.* 2018 showed that serum concentrations of asprosin were positively associated with LDL-C, apoB and apoE [21].

We did not observe any significant difference in lipid profile as well as asprosin concentration between male and female newborns. However, a study by Kelishadi et al*.* 2007 reported that total and HDL cholesterol in girls were significantly higher than in boys [9]. Moreover, a study by Ghiasi et al*.* 2013 reported that the cord blood from female newborns had higher levels of LDL-C, HDL-C and total cholesterol compared to male newborns [22]. Furthermore, Jahanfar et al*.* 2016 in a cohort study of twins, reported that male-male twins were heavier than male-females and female-female twin pairs [23].

Our study found a positive but non-significant association between asprosin concentration and anthropometric indices. A study by Hoffmann et al*.* 2022 on 247 umbilical plasma samples reported that there was no significant correlation between BW and BL with asprosin concentration [24].

### Biological plausibility

Asprosin may affect lipid metabolism by two different mechanisms: the effect on the insulin signaling pathway and proopiomelanocortin (POMC)-positive neurons activity. Some effects of asprosin on lipid profile may be exerted by altering gene expression in liver cells through insulin resistance induction [25–28]. High insulin concentrations in IR alter the expression of some genes [29–32]. In the liver, the target tissue of asprosin, insulin induces the expression and activation of enzymes involved in hepatic lipid production [33–37]. Although the molecular mechanism of asprosin on insulin singling is not well known; however, several studies suggested elevated concentrations of asprosin interfere with insulin function and induces insulin resistance [38–41]. Romere et al. 2016 showed that single injection of asprosin results in hyperglycemia and hyperinsulinemia [14]. Wang et al*.* 2018 found a negative relationship between serum asprosin concentrations and indicators regarding the first-phase insulin secretion, such as AUC, AIR, and GDI and HOMA-β, and a positive correlation with HOMA-IR [20]. They suggested that the asprosin-related metabolic pathways dysregulation might be through its role in ꞵ-cell dysfunction and insulin resistance [20]. Jung et al*.* 2019 showed that treatment of skeletal muscle cells by recombinant asprosin results in impairment of insulin sensitivity through PKCδ-associated ER stress/inflammation pathways [26]. Lee et al. 2019 showed that treatment of primary human islets with recombinant asprosin induced the inflammation response, cellular dysfunction, and apoptosis in a dose-dependent manner [42].

Asprosin exerts some of its effects by changing the function of the CNS system. Duerrschmid et al*.* 2017 demonstrate that asprosin in the circulation crosses the blood–brain barrier and inhibits the downstream anorexigenic proopiomelanocortin (POMC)-positive neurons. The inhibition of these neurons leads to appetite stimulation and a drive to accumulate adiposity and body weight [19, 43, 44]. Blockade of the CNS melanocortin system increased triglyceride synthesis in the periphery and triglyceride content in the liver [45, 46].

### Limitations

Our study has some limitations that should be considered in future studies. The sample size was relatively limited, and the findings of this study required to confirm from other ethnicities. Also, the cross-sectional nature of this study did not allow us to address the underlying signaling pathways. Moreover, we did not have any data on pre-pregnancy lipid profile, maternal diet, maternal weight gain and other prevalent endocrine disorders like PCOS that can affect our results. Furthermore, we missed data about timing of cord clamping that could affect TG and total cholesterol. Research in cellular models is required to determine underlying mechanisms.

## Conclusion

The present study indicated that asprosin concentration in umbilical cord blood was positively associated with TAG, TC, LDL-C concentration and TAG/HDL-C, TC/HDL-C, LDL-C/HDL-C and non-HDL-C/HDL-C ratio. Our data provide new clinical information about the role of adipokines in the regulation of atherogenic lipids including TC and LDL-C in umbilical cord blood. Further studies including the identification of the molecular changes in tissue structure or functions, are needed for a better understanding of asprosin- lipid profile and its clinical outputs in humans.

## Data Availability

The data that support the findings of this study are available from the corresponding author upon reasonable request.
